# Research on Material Design of Medical Products for Elderly Families Based on Artificial Intelligence

This article has been retracted.

**DOI:** 10.1155/2022/7058477

**Published:** 2022-01-18

**Authors:** Jinjin Rong, Xu Ji, Xin Fang, Moon-Hwan Jee

**Affiliations:** ^1^Department of Convergence Design, Hanseo University, Seosan, 31962 Chungcheongnam-do, Republic of Korea; ^2^School of Art, Anhui University of Finance and Economics, Bengbu, 233000 Anhui, China; ^3^College of Fine Arts, Anhui Normal University, Wuhu, 241002 Anhui, China

## Abstract

Due to the rapid growth of the elderly around the world, the artificial intelligence control framework can collect information and apply it and perform other tasks. Artificial intelligence plays an important role in focusing on the elderly. For example, it can improve the relationship between the elderly and family members or nursing teams. In addition, AI chat robot can communicate with the elderly without obstacles and can remind the elderly when to take medicine, regular physical examination, etc. A significant number of the AI applications on cell phones accessible today could screen wellbeing information, like every day exercises, diet, and surprisingly the senior's way of life, in a less nosy way. In such cases, it could help in expecting and, subsequently, forestalling any conceivable hypertension or unpredictable heart rate. Essentially, mechanical ‘pets' are likewise assisting with fighting off feelings of loneliness, while additionally assisting with upgrading patient consideration simultaneously. One model is Tombot, a little dog like model, which was made to diminish misery and tension among dementia patients. Its head developments, looks, and swaying tail feel basically the same as the real thing, causing occupants to feel as though they have their very own pet to really focus on. One of the issues that growing societies are presently facing is the care of elderly individuals. The dearth of skilled workers in the senior healthcare setting has been exacerbated by the worldwide shift of aging populations. There might be an enhanced need for old nursing since the global older demographic is expected to nearly triple in the coming three decades. There are advancements in computer technologies for supporting the aged plus associated caregivers, checking their wellbeing, and offering company to them. Given the global elderly demographic development possibilities, it is no coincidence that the aided care market is drawing fast advancement, rendering health management for nurses a breeze. While the world's governments manage the aging population next years, these ideas will become extremely vital. They will almost certainly encounter economic and political demands to modify state medical care management, retirement benefits, and social security in order to meet the needs of an aging population. Considering that the demand for physicians is growing, a necessity has developed to deliver individualized care for the aged as well as to respond appropriately in emergencies. As a result, in the technological society, healthcare is exploring artificial intelligence to deliver personalized treatment to individuals in need. The challenges of the aged are determined in this study, and answers are supplied via a tailored computer (robot). With the crucial details given via Internet of Things gadgets, emergency events may be foreseen relatively promptly, and appropriate actions can be proposed by AI technology. Individuals' vital health information is collected using the Internet of Things based on smart technology. The information is evaluated, and decisions are made by AI, while the developed machine performs the appropriate task. This research, therefore, looks at the material design of medical products for elderly people based on artificial intelligence. It goes further and explains some of the challenges encountered in the process and possible remedies.

## 1. Background

The employment of artificial intelligence technology in healthcare has been discussed since the dawn of the contemporary age. This is unsurprising, given that AI technologies are designed to mimic the real person's brain's functionality. “Computer technology would certainly exercise its greatest influence by supplementing and, for other circumstances, substantially substituting the cognitive tasks of the doctor,” remarked William B Schwartz, a doctor intrigued by the application of computer technology in medicine, in 1970. Towards the 1970s, it was clear that traditional computational approaches proved inadequate for dealing with complicated healthcare issues. For medical decision-making, a rather advanced digital system that emulated human reasoning, i.e., an artificial intelligence-based system, was necessary [1]. The first attempts to use AI in healthcare were to establish rule-based systems to assist with clinical thinking. Severe medical challenges, on the other hand, are far too sophisticated to be solved using basic rule-based problem resolution strategies. The design of computer algorithms related to illness concepts preceded problem-solving in healthcare [2]. AI was being used to help with resolving challenges in a variety of fields, not only basic healthcare. Gunn, a Scottish surgeon, pioneered the application of numerical simulations to identify severe abdominal discomfort in 1976. Medical inspections of organized patient records via computer systems were used to accomplish this, with a diagnosis under this way proving to be roughly 10% greater inaccuracy than the usual approach. Around the 1980s, artificial intelligence study organizations had found themselves all over the globe, but particularly at educational centers. This advancement aided the spread of new and creative AI techniques to clinical diagnosis. Healthcare was a great experimental environment for the latest AI technologies; therefore, there were a lot of purchases behind it. During this point, the expert system approach was used in a substantial percentage of AI applications in medicine. Clinical cognitive computing had begun to apply modern tactics such as machine learning and convolutional neural networks to improve medical discernment call through the conclusion of the 20th century.

### 1.1. Introduction

Now, how exactly do we explain artificial intelligence? There exist various definitions of what artificial intelligence is and what goes into producing AI due to the sophistication needed in generating artificial intelligence that is equivalent to that of human nature.

In societies, computers are directing choices about elder care, driven by lack of caregivers, an aging population, and wanting their seniors to stay in their own homes longer. Plenty of so-called ‘age tech' companies have come up over the last few years to keep tabs on older adults, particularly those with cognitive decline. Their solutions are now beginning to permeate into home care, assisted living and nursing facilities.

Organizations like Apple and Fitbit have made smart wearable biometric trackers accessible to a huge segment, including old and geriatric patients. Older patients can utilize this current gadget's implicit AI-controlled usefulness to really take a look at irregularities in their biometric information, just as to recognize a critical or hard fall and sound a caution. AI Care professes to utilize AI examination and wearable sensor to customize the consideration for every older customer [3].

The innovation can free up human caregivers so they can be as proficient as potentially possible. Essentially, mechanical ‘pets' are likewise assisting with fighting off feelings of loneliness, while additionally assisting with upgrading patient consideration simultaneously [4]. One model is Tombot, a little dog like model, which was made to diminish misery and tension among dementia patients. Its head developments, looks, and swaying tail feel basically the same as the real thing, causing occupants to feel as though they have their very own pet to really focus on.

Other writers despise the phrase artificial intelligence and choose to use the phrase computational intelligence instead. Nevertheless, if we evaluate what artificial intelligence's goal is and what tools are used to achieve it, we may come up with an appropriate description that includes all of these elements. The ultimate goal of artificial intelligence is to construct machines that process information intelligently in the same way that people do [5]. Intelligent agents are another title for these technologies [6].

If the objective of this model is to illustrate intelligence, and constructing such frameworks necessitates computer programming, a structured description of artificial intelligence would be stated as a domain of scientific knowledge involved with the computational understanding of what is frequently referred to as intelligent behavior [7], as well as the development of intelligent agents that display such behavior. Relatively simplified descriptions of artificial intelligence include devices that mimic human functionalities [8], the expansion of human intelligence via machines, and programming computers to perform tasks that humans now perform, though a truer definition would have been the science of creating smart machines [9].

### 1.2. The Smart Machine Concept

The smart agent (Figure 1) notion is the clearest way to understand artificial intelligence theory. A smart agent possesses the abilities necessary to satisfy the Turing Test, which determines for certain if or not a computer can reason like a person. As a result, a smart agent ought to be capable of sensing, realistic judgment, and response to fulfill its objectives. To both take input and perform reactions, the device makes use of the surroundings in which it functions. Present perceptions about the surroundings, preexisting information about the surroundings, histories through which it can learn, and the goals it intends to attain are among the primary inputs that enter into the device and possibly which it can extract independently [10]. The device uses electronic sensory detectors to assess the surroundings and signaling pathways to interact with it. A ‘robot' is a smart device that combines a computer foundation with mechanical actuators and sensors [11]. An ‘infobot' is software that acts in a refined algorithmic context, but a judgment assistance technology is a program that provides guidance and is paired with a human operator.

### 1.3. Constituents of an Artificial Intelligence Technology System

Intelligence is defined by the ability to acquire knowledge. Learning entails gaining additional knowledge, acquiring additional abilities via teaching or practice, and representing and experimenting with that awareness. If artificial intelligence includes the acquisition of knowledge, it must exhibit all of the previously stated characteristics. Machine learning is a typical method for AI technologies to fulfill their learning aims [12]. Machine learning is the computerized modeling of various components of the process of acquisition of knowledge. The ability of algorithms to self-learn and develop via practice is one of the most important aims of machine learning. There are two types of ML algorithms: monitored and unmonitored. An algorithm operating with tagged instructional information is used in monitored training. Monitored training involves information categorization and programming of the link across incoming and end data. Unmonitored learning, on the other hand, permits an algorithm to find a concealed trend in a set of data. In this, the algorithm is used to see what trends can be found in the information and what possible results may be predicted [13].

With AI, the thought is that PCs learn by taking in data. As they see and experience more data, they get more intelligent. Be that as it may, the same old problem exists. They should comprehend the data they are being shown to appreciate precisely what it is and its importance to what they definitely know.

For example, it is helpful to perceive that a vehicle has driven past the road. Simply while having the option to distinguish a vehicle with a driver inside—rather than it being some other item moving past the visual edge like a bird—would AI be able to begin to see the value in addition with regard to it. When it knows it is a vehicle, it can gauge speed and decide if the vehicle is going quicker than the allowed speed limit [14].

It might likewise draw an association between the vehicle, its tag, and the record of the proprietor of that vehicle. While these things can be caught autonomously, having the option to arrange the data with the AI what is important and what is not is something amazing.

Previously, researchers hoped that artificial intelligence might be able to imitate people's cognitive abilities. This method has been known as “Traditional AI.” This was, unfortunately, a restrictive method because it supposed that human intellect was the sole source of cognition. This method also presupposes that human intellect is the highest level of intelligence possible. Learning and thinking are the two basic components of intelligence. The constraints of human intellect do not have to restrict how the intellect is constructed. The illustration of flight is a good one to use in this context. While bird flight might serve as a form of motivation for aircraft design, the architecture of an aircraft does not replicate the physical anatomy of a bird. As a result, it is far more crucial to add critical intelligence features into artificial intelligence as opposed to simply copying human intellect.

Additional parts of artificial intelligence and machine learnings are cognition and knowledge organization. Within artificial intelligence technology, logical thinking entails manipulating facts to generate responses. Contrasting it to conventional programming, AI focuses on what needs to be processed rather than how it needs to be processed. Design-time logic, offline calculation, and online calculation are used to structure this processing. Algorithms centered on the step-by-step logic approach were employed to solve predicted issues in previous kinds of AI. Such systems, on the other hand, proved useless in unclear circumstances or when there was insufficient data. To react to such circumstances, artificial intelligence-based logic systems have been developed to incorporate elements from statistical and economic concepts. AI technologies need extensive awareness of the appropriate surroundings, as well as the ability to encode this knowledge in a mathematical format to address challenges, whether they are predictable or unpredictable. AI employs a Representation and Reasoning System (RRS) to do this. The RRS consists of a programming language for communicating with a computer, a mechanism for allocating significance to the code, and a method for determining the replies following input. Information can be expressed in a variety of ways, though the most common form is Frames.

Programming languages and computing materials constitute 2 fundamental features that permit artificial intelligence-based knowledge expression and thinking. Multiple programming languages are employed in artificial intelligence technology. Low-level programming languages like Lisp, Python, C++, and Fortran are the majority. Over the years, the growth of artificial intelligence technology was hampered by self-contained computers and their constrained computational capability.

### 1.4. AI Devices

Essentially, there exist 2 sorts of artificial intelligence machines: the first is the machine learning division, which analyzes structured data such as electrophysiological information, genetic information, and image analysis information. Machine learning systems in medical solutions attempt to collect patient distinctiveness or comprehend the probability of illness impacts [15]. Natural language processing technology is the next sort of AI device, and it may extract data from unconstrained or unorganized information such as clinical inspections or medical records in order to improve formatted medical screening information. NLP transforms items into machine-understandable organized files, which could subsequently be explored by computer learning techniques. The diagram below depicts the path from medical data creation to clinical decision creation (Figure 2), including NLP information enhancement and machine learning information analysis. The route map in this diagram begins and concludes with healthcare activity. As powerful as AI techniques are, they can be motivated by healthcare issues and also be useful in improving clinical competence.

## 2. Process of Machine Learning (ML)

Machine learning creates a data-mining set of rules that extract features from the information. Patient's ‘characters' moreover on rare occasions, treatment outcomes of interest are used as inputs to a machine learning set of rules. Important data, such as sexual identity, age, clinical background, disease exact data, such as gene expressions, analytical imaging, electrophysiological data test, objective diagnostic studies, medicine, and clinical signs, are commonly found in a patient's characters. Clinical findings are frequently generated for clinical examination in conjunction with the patient's characteristics.

*Pij* represents the *j*th feature of the *i*th actual figures of patients, and *Qi* represents the impact of interest. The ML set of rules can also be divided into 2 sorts based on whether or not the findings should be integrated: monitored training and unmonitored training. There is also a sort of training known as semisupervised training. All 3 forms of learning approaches are depicted in the diagram below (Figure 3).

Monitored training is suitable for statistical modeling by establishing multiple relationships connecting patient uniqueness (input) as well as the outcome of interest, while unmonitored training is useful for attribute elimination (output). Semimonitored training has recently been shown as a combination of monitored and unmonitored training that is ideal for situations when the impact is excluded for certain reasons.

### 2.1. The Neural Network

A neural network can be referred to as a type of regression analysis that has been used to confine problematic complex interactions by splitting the input variables and output information. The relationships between the intake variables and the results are expressed in this neural network by many unidentified strata clustering of preindividual functions. The goal is to estimate the balances using information and result information, reducing the mean inaccuracy associated with the result and its computation. This approach is explained below with the help of a few illustrations as shown. Some entry variables for the neural network in ictus diagnosis were *Xi*1, ⋯*Xip* and *p* = 16 ictus-related indicators, such as severe disorientation, visual and movement problems, and leg or arm numbness or tingling. *Yi* denotes a binary result, with *Yi* = 1/0 indicating whether the *i*th individual has or has never had ictus. The important output component is the ictus likelihood *ai*, which is represented by the formula that follows (Figure 4).

*Xij*, fk = 0; *fks* as well as *h* are predefined functions, and w10 and w20 are not equivalent to 0 in this formula, indicating that the proportional clustering affects the illness danger entirely. The neural network technology is depicted in the diagram below Figure 5.

### 2.2. Remedies for Physical Challenges

One primary goal of robotics and artificial intelligence is to help the aged in undertaking daily duties while assuring their safety at their residences. Automated vacuum cleaners, coffee makers and cutlery, lawnmower, washing machines, and food warming appliances are just a few of the robotic items. Humanoid robots, prosthetic appendages, and smart wheelchairs are among the contemporary robotic applications. Bots have also been created to hoist or support humans, and robotic walkers are now being designed for individuals that move with a walking stick; for instance, Dublin scientists produced a personal mobility device that can be managed similar to a smart walker (Table 1).

Around 2004, a concept of a computer-controlled walker called Guido was constructed for the partially sighted that could assist the aged in navigating by relaying data regarding their environment and adjacent items. Pearl and Care-O-bot, as well as AILISA, were also examples of the bots presently in construction. Pearl can keep track of a client's healthcare, communicate with them, and notify them of their meetings. Care-O-bot can keep track of your wellbeing, regulate your home surveillance, use the microwave, get items, and contact family and medical specialists. AILISA keeps track of the client's accidents and physiological complaints.

Bots are also being created to assist aged people with regular tasks which include showering. The Harmony in Roll-lo Bathing (HIRB) robotic device is an example of a robot that assists the aged in showering. A user takes a seat on a seat that rolls backward into a compartment that completely covers their torso, keeping the shoulders as well as head outside the compartment. This bot is again programmed to discharge body wash and water into the compartment, allowing the human to be bathed. The above bot is currently getting evaluated in Japan, and the results are promising. Humans' confidentiality and privacy are supposed to be protected by these bots, which are also simpler to operate and save time [16]. Showering is among the most challenging duties for the aged, so these bots could come in handy. They can also be used to substitute showers, reducing the chance of falling in the restroom.

### 2.3. Remedies to Cognitive Challenges

Embedded software in bots serves to exercise the mind through mental practice sessions. Cafero is a bot that supervises wellness, offers telecommunications solutions, and gives cognitive instruction. The bot has been put to the test in dementia centers and care facilities. Bots that give exercises for cognitive stimulation, musical treatment, and reminiscence treatment are intended specifically for dementia clients [17]. Such individuals are constantly stimulated and occupied in order to reduce their disruptive habits, lowering nurse frustration and enhancing patient integrity of existence.

Infobot and IRobiQ are bots designed to deliver cognitive activities and a variety of additional applications. Regarding dementia sufferers, specialists recommend these bots have embedded software. As a result, such bots can stimulate cognitive brain exercise routines while simultaneously measuring and monitoring their physical well-being.

## 3. Conclusion

This study looked at the things society needs to ensure that the aged can remain autonomous in their households under the assistance of bots. With the advancement of automation in the realm of medicine, such demands will remain to be met. This study demonstrated how the aged require assistance with day-to-day tasks and physical activity. As individuals get older, particularly as they stay on their own, accidents and injuries become more of a worry. Individuals become forgetful as they age and may need official assistance. The aged also have a lot of medical issues and mental impairments, so it is necessary to keep track of their overall health and manage their health problems. Although the aged are capable of dealing with the obstacles of aging, they could become unhappy, secluded, and lonesome. Furthermore, owing to an increase in the demand for physicians, primarily because of contagious infections such as the coronavirus, necessity has developed to deliver tailored care for aged individuals and those suffering chronic problems, as well as to respond appropriately in an emergency. As a result, IoT peripheral gadgets are employed to collect vital clinical information from patients. Artificial intelligence processes the data and makes decisions, while the necessary operation is performed by a robot created specifically for the task. The bots will be designed to avoid assistance, execute numerous operations, create motivated connections, save more academic information, and notify an ambulance in the event of an incident.

## Figures and Tables

**Figure 1:** Smart agent concept.

**Figure 2:** Plan for medical data generation.

**Figure 3:** (a) Monitored, (b) unmonitored, and (c) semimonitored.

**Figure 4:** Approach.

**Figure 5:** Neural network illustration.

**Table 1:** Examples of conditions assisted with bots.

Issues faced by the elderly	Current solutions	Robots that can solve issues
Medications and health management	Memory device [13], personal digital assistant(PDA), medicine dosage regimes [14]	Hector [15], Care-O-bot [16], Teddy [17], Wakamaru [18], IRobiQ [19]
Mobility for the physically disabled	Walking stick, wheelchair, mobility scooters, and transportation services	Guido [20] and robotic wheelchairs [21]

## Data Availability

The data underlying the results presented in the study are available within the manuscript.
